The article "Repeat Confirmatory Testing for Persons with Discordant Whole Blood and Oral Fluid Rapid HIV Test Results: Findings from Post Marketing Surveillance" was published in 2008. Journal: PLoS One.

# Repeat Confirmatory Testing for Persons with Discordant Whole Blood and Oral Fluid Rapid HIV Test Results: Findings from Post Marketing Surveillance

**DOI:** 10.1371/journal.pone.0001524

**Published:** 2008-02-06

**Authors:** Laura G. Wesolowski, Duncan A. MacKellar, Steven F. Ethridge, Julia H. Zhu, S. Michele Owen, Patrick S. Sullivan, for the Post Marketing Surveillance Team

**Affiliations:** Division of HIV/AIDS Prevention, National Center for HIV, STD and TB Prevention, Centers for Disease Control and Prevention, Atlanta, Georgia, United States of America; Medical Research Council South Africa, South Africa

## Abstract

**Background:**

Reactive oral fluid and whole blood rapid HIV tests must be followed with a confirmatory test (Western blot (WB), immunofluorescent assay (IFA) or approved nucleic acid amplification test (NAAT)). When the confirmatory result is negative or indeterminate (i.e. discordant with rapid result), repeat confirmatory testing should be conducted using a follow-up specimen. Previous reports have not described whether repeat testing adequately resolves the HIV-infection status of persons with discordant results.

**Methodology:**

Post-marketing surveillance was conducted in 368 testing sites affiliated with 14 state and 2 city health departments from August 11, 2004 to June 30, 2005 and one health department through December 31, 2005. For persons with discordant results, data were collected on demographics, risk behaviors, HIV test results and specimen types. Persons with repeat confirmatory results were classified as HIV-infected or uninfected. Regression models were created to assess risk factors for not having repeat testing.

**Principal Findings:**

Of 167,371 rapid tests conducted, 2589 (1.6%) were reactive: of these, 2417 (93%) had positive WB/IFA, 172 (7%) had negative or indeterminate WB/IFA. Of 89/172 (52%) persons with a repeat confirmatory test: 17 (19%) were HIV-infected, including 3 with indeterminate WB and positive NAAT; 72 (81%) were uninfected, including 12 with repeat indeterminate WB. Factors associated with HIV-infection included having an initial indeterminate WB/IFA (vs. negative) (p<0.001) and having an initial oral fluid WB (vs. serum) (p<0.001). Persons who had male-female sex (vs. male-male sex) were at increased risk for not having a repeat test [adjusted OR 2.6, 95% CI (1.3, 4.9)].

**Conclusions:**

Though only half of persons with discordant results had repeat confirmatory testing, of those who did, nearly one in five were HIV-infected. These findings underscore the need for rapid HIV testing programs to increase repeat confirmatory testing for persons with discordant results. Because of the lower sensitivity of oral fluid WBs, confirmatory testing following a reactive rapid test should be conducted using serum or plasma, when possible.

## Introduction

The OraQuick Rapid HIV Antibody Test (OraQuick) was the first HIV rapid test to be approved by the Food and Drug Administration (November 2002) and to be waived under the Clinical Laboratory Improvement Amendments of 1988 (CLIA) (February 2003) for use at point of care [1], [2]. The Centers for Disease Control and Prevention (CDC) initiated surveillance to assess the accuracy of waived rapid HIV testing. The OraQuick test performs within the manufacturer's claim with few false positives when used on whole blood (specificity 99.90% to 99.98%) and oral fluid (specificity 99.60% to 99.89%), though clusters of false positives and false negatives may occur [3]–[8]. HIV prevalence in the population being tested can affect test performance, particularly positive predictive value, the probability that a person actually has HIV given that he or she tests positive [7]. Per the manufacturer's instructions, the rapid test is typically run in singlet [3], and all reactive (preliminary positive) rapid test results should be confirmed with either a WB, IFA, or approved NAAT test [9]. In cases where the confirmatory test result is discordant with the reactive rapid test result (i.e., the WB or IFA is negative or indeterminate), a repeat confirmatory test should be performed on a new follow-up specimen [9], [10].

Repeat confirmatory testing is important to rule out labeling or laboratory error as the reason for the discordant test result. It is also needed if the screening test is more sensitive than the supplemental test used to confirm infection. Differences in sensitivity between the screening and confirmatory tests may be particularly important for programs that use a rapid test on whole blood for screening and a WB on oral fluid for confirmation. Compared with assays performed on whole blood, serum, or plasma, assays performed on oral fluid have a lower sensitivity due to the lower antibody concentration found in oral fluid [11]–[14]. Therefore, a blood specimen obtained during a follow-up visit is recommended for repeat confirmatory testing for persons who have a preliminary positive rapid test result followed by an initial confirmatory test result that is not positive [9], [10].

Since the widespread use of rapid tests began in publicly funded HIV test programs in 2003, no reports have described (1) whether current testing guidelines for repeat confirmatory testing are adequate for resolving the infection status of clients with discordant test results and (2) the magnitude and correlates of not having repeat confirmatory testing among persons with discordant HIV test results [15]. One report with a small number of discordant cases characterized the infection status of persons with discordant results who had repeat confirmatory testing but did not examine correlates of not having repeat testing [10]. Information on whether HIV infection status is resolved for persons with initially discordant test results who adhere to guidelines for repeat confirmatory testing is important for guiding public health rapid HIV test programs, especially those that use oral fluid for initial WB confirmation and those that have experienced excessive discordant test results [4]–[7].

This report uses data obtained from CDC's Post Marketing Surveillance Program to evaluate the HIV infection status of persons with reactive rapid HIV results and discordant confirmatory test results who have repeat confirmatory testing. We also assess the magnitude and correlates of not having repeat testing.

## Methods

### Surveillance System

Rapid test post marketing surveillance was conducted in 368 rapid HIV test sites affiliated with 14 state (Arizona, Delaware, Florida, Indiana, Louisiana, Massachusetts, Michigan, Montana, Nebraska, New Jersey, New York, North Carolina, Utah, Wisconsin) and 3 city (Chicago, New York City, San Francisco) health departments from August 11, 2004 to June 30, 2005. These health departments were chosen based on their applications to CDC in which they demonstrated their ability to conduct rapid testing. Surveillance continued in one city health department through December 31, 2005 in response to a cluster of false-positive rapid test results at one test site [7]. Health departments selected rapid test sites within their jurisdiction to participate in surveillance. Whole blood (collected by fingerstick and venipuncture) and oral fluid rapid tests routinely conducted at each site were included in surveillance. Although all health departments, except three (Delaware, Massachusetts, and Montana), offered whole blood and oral fluid rapid tests in at least one of their sites during surveillance, information on whether each person tested was offered both whole blood and oral fluid rapid testing was not collected on a case-by-case basis. Post marketing surveillance was determined not to be research by CDC since it consisted of routine public health disease surveillance, and therefore Institutional Review Board approval was not required by CDC.

Oral fluid or blood specimens from clients with reactive rapid tests were submitted to local laboratories for enzyme immunoassay (EIA) screening (optional) followed by WB or IFA confirmation (initial confirmatory testing). CDC recommended that all persons with discordant results return for repeat confirmatory testing, preferably with a blood specimen [9], [10]. Local laboratories used FDA-approved EIA, WB, IFA and nucleic acid amplification (NAAT) tests in accordance with local procedures. For all persons with a reactive rapid test result followed by a negative or indeterminate confirmatory test, case report forms which included information on patient demographics, HIV risk behaviors, and initial and repeat HIV test results were completed and submitted to CDC. Two health departments collected data on the appearance of test lines on rapid test devices that produced discordant test results from January 1, 2005 to June 30, 2005. Affiliated laboratories of participating health departments sent to CDC available remnant serum or plasma from initial or repeat specimens collected from persons with discordant rapid test results. Remnant oral fluid specimens were not submitted because they cannot be stored as long or undergo as many freeze-thaw cycles as blood or plasma [11]. From September to November 2005, interviews were conducted with principal investigators from participating health departments to assess the completeness of discordant case reporting and to assess reasons for not obtaining repeat confirmatory specimens.

At CDC, remnant serum was tested by the third-generation Genetic Systems HIV-1/HIV-2 Plus O EIA, and Calypte HIV-1 or Genetic Systems HIV-1 WB. Western blot tests were run at CDC even if an EIA was negative. If remnant plasma was sent, it was tested individually using the Roche Cobas Amplicor HIV-1 Monitor Assay. If plasma was not sent, a qualitative NAAT for HIV-1 RNA (Gen-Probe Procleix HIV-1 RNA Assay) was run off-label on remnant sera. HIV RNA detection using Gen-Probe Procleix HIV-1 RNA Assay was performed in pools of up to 16 serum specimens.

### Analyses

To evaluate the infection status of those who underwent repeat confirmatory testing, we classified persons as: (1) uninfected (false positive rapid test result) if the last repeat EIA was negative (if performed) and the last repeat WB or IFA was negative or indeterminate, and HIV-1 RNA was not detected in any initial or repeat confirmatory specimens if tested with NAAT; and (2) infected (true positive rapid test result), if the WB conducted at CDC on an initial or repeat confirmatory specimen was positive or if the IFA or WB conducted on a repeat confirmatory specimen at the participating laboratory was positive, or if HIV-1 RNA was detected at a local laboratory or at CDC on either the initial or repeat confirmatory specimen. Since indeterminate Western blot test results can occur in uninfected persons, we chose to classify as not infected those persons whose repeat confirmatory WB or IFA test was indeterminate provided other serologic or nucleic acid tests did not suggest infection [16], [17]. For HIV-1 uninfected and infected, we report the type of initial and repeat confirmatory specimens that were obtained; available initial and repeat confirmatory serologic and nucleic acid test results; and the interval in days from the initial confirmatory test to the last repeat confirmatory test for persons classified as not infected, and first positive confirmatory test for persons classified as infected. We also report available test line appearance for rapid test devices of persons with discordant test results.

In univariate analyses, we used Mantel-Haenszel chi square tests and odds ratios with 95% confidence intervals to assess demographic, behavioral, and initial testing correlates of not having repeat confirmatory testing. Effect modification was assessed using the Breslow Day test. Variables which were associated (p<0.2) with not having repeat confirmatory testing in univariate analysis were included in the multivariate logistic regression model. Goodness of fit was assessed using the likelihood ratio test. Analyses were performed using SAS version 9.1 (SAS Institute, Cary, North Carolina, USA).

## Results

There were 167,371 rapid tests (136,798 whole blood and 30,573 oral fluid) conducted during the post marketing surveillance period, including the extended surveillance in one health department. There were 2589 (1.6%) reactive rapid tests; of these, 2417 (93%) had confirmatory test results that were positive (2033 whole blood rapid, 384 oral fluid rapid) and 172 (7%) had confirmatory test results that were negative or indeterminate (72 whole blood rapid and 100 oral fluid rapid). Of the 172 persons with discordant test results, 74% were male; 50% were 33 years old or younger (range 15 to 82); 45% were white, non-Hispanic, 31% were black, non-Hispanic, 10% were other race, non-Hispanic, and 13% were Hispanic. The gender, age and race of persons presenting for rapid testing at all post marketing surveillance sites were described previously [7].

### Repeat Confirmatory Practices and HIV-1 Infection Outcomes

#### Testing practices

Of the 172 persons with discordant test results, 89 (52%) had ≥1 repeat confirmatory tests conducted and 83 (48%) did not have repeat testing (Figure 1). Overall, 83 (93%) of 89 persons with a repeat confirmatory test had a repeat confirmatory test performed on a serum specimen, including 18 whose initial confirmatory test was conducted using oral fluid (Figure 1).

**Figure 1:** Repeat confirmatory testing practices after a reactive rapid HIV test and negative or indeterminate WB/IFA. WB = Western blot, IFA = Immunofluorescent assay, OF = oral fluid, IND = indeterminate, NEG = negative.

Of the 83 persons on whom a repeat confirmatory test was *not* done, most 66 (80%) had an initial confirmatory WB/IFA performed on serum, including 1 initial indeterminate which was classified as Western blot positive at CDC. With the exception of that individual, the HIV-infection status of these persons is not known.

#### Repeat testing HIV-1 infection outcomes

Of the 89 persons with a discordant confirmatory test result on whom ≥1 repeat confirmatory tests were conducted, 72 (81%) were classified as uninfected (false-positive rapid test result) and 17 (19%) were classified as HIV-1 infected (true-positive rapid test result). Those whose initial confirmatory WB/IFA result was indeterminate were more likely to be HIV-infected (15/24 63%) compared with those whose initial confirmatory WB/IFA result was negative (2/65 3%) (p<0.001). Those whose initial confirmatory test was conducted on oral fluid were more likely to be HIV-infected based on repeat confirmatory testing (13/23 57%) compared with those whose initial confirmatory test was conducted on serum (2/64 3%) (p<0.001). The association between initial confirmatory specimen type and follow-up HIV-infection status remained statistically significant when stratified by whether initial confirmatory test result was negative or indeterminate (data not shown).

#### HIV-1 uninfected (False-positive rapid test)

Of the 72 persons classified as uninfected, 29 (40%) had a whole blood rapid test and 43 (60%) had an oral fluid rapid test.

Of the 60 persons classified as uninfected whose repeat WB/IFA test result was negative, 57 (95%) had EIAs performed at the local laboratory on the initial confirmatory specimen, and of these, 1 (2%) was reactive; 47 (78%) had EIAs performed on the repeat confirmatory specimen at the local laboratory, and of these, 1 (2%) was repeatedly reactive. For these 60 uninfected persons, the median interval in days between the initial confirmatory test and the last repeat negative confirmatory test was 36 (range: 6-235). Of these 60, 23/23 (100%) had undetectable virus based on Procleix testing on remnant serum, including 12 who had a short interval between initial confirmatory test and last repeat negative confirmatory test (< = 36 days).

Of the 12 persons classified as uninfected who had a repeat confirmatory WB test result that was indeterminate, 12/12 (100%) had a repeat negative EIA at the local laboratory, 8/9 (89%) had a repeat negative EIA at CDC, 6/6 (100%) had a repeat negative IFA, and 7/7 (100%) had a negative NAAT result on either the initial or repeat confirmatory specimen or both (Table 1). The median interval between the initial confirmatory test and the last repeat indeterminate WB for these 12 persons was 24 days (range: 7–81 days). Of the 7 persons with negative NAAT results, 3 had a short interval between initial confirmatory test and last repeat negative confirmatory tests (< = 24 days).

**Table 1:** Test results for 12 persons with reactive rapid test results classified as HIV-uninfected but who had an indeterminate WB at the last repeat confirmatory test, 17 health departments, 11 August 2004 to 31 December 2005.

	Initial Discordant Test Results					Last Repeat Confirmatory Test Results					
OraQuick specimen type	Confirmatory specimen type	EIA	WB Bands	IFA^b^	NAAT	Days after first confirmatory test	Confirmatory specimen type	EIA	WB Bands	IFA^b^	NAAT
Oral	Serum	Neg^a^ [Neg]	[p24*, p55]	Neg	[Neg]^c^	7	Serum	Neg^a^	[p24* ]	Neg	[Neg]^d^
Oral	Serum	Neg^e^	p24^f^	ND	ND	11	Serum	Neg^e^	p24^f^	ND	ND
Oral	Serum	Neg^a^ [Neg]	[p24, p55*]	Neg	[Neg]^c^	19	Serum	Neg^a^ [Neg]	[p24*]	Neg	[Neg]^d^
Oral	Serum	Neg^a^ [Neg]	[p24]	Neg	[Neg]^c^	22	Serum	Neg^a^ [Neg]	[p24]	Neg	[Neg]^c^
Oral	Serum	Neg^a^ [Neg]	[p18, p55*]	Neg	[Neg]^c^	26	Serum	Neg^a^ [Neg]	[p18*]	Neg	[Neg]^d^
Oral	Serum	Neg^a^ [Neg]	[p24, gp41, p55]	Neg	[Neg]^c^	34	Serum	Neg^a^ [Neg]	[p24, p55]	Neg	[Neg]^c^
Oral	Serum	Neg^g^	p51, p66 h [p51, p65]	ND	ND	49	Serum	Neg^g^ [Neg]	p17, p24, p55, p66 h [51, 65]	ND	ND
Oral	Serum	Neg^a^ [Pos]	[p24]	Neg	[Neg]^c^	81	Serum	Neg^a^ [Pos]	[p24*]	Neg	[Neg]^d^
Blood	Oral	Neg^a^	None^i^	ND	ND	19	Serum	Neg^g^ [Neg]	None^h^ [p66, p31]^h^	ND	ND
Blood	Oral	Neg^a^	None^i^	ND	ND	21	Oral	Neg^a^	p24^i^	ND	ND
Blood	Serum	Neg^a^	p17^f^ [p17]^h^	ND	ND	28	Serum	Neg^a^ [Neg]	p17^f^ [p17]^h^	ND	[Neg]^d^
Blood	Serum	Neg^g^ [Neg]	p66^h^ [p66]^h^	ND	ND	29	Serum	Neg^g^ [Neg]	p66^h^ [p66]^h^	ND	ND

EIA = enzyme immunoassay, WB = Western blot, Neg = Negative, ND = Not done *Bands interpreted as equivocal

[ ] results reported by CDC lab where Genetic Systems HIV1/HIV2 Plus O and Genetic Systems HIV-1 Western blot were used unless otherwise noted

a Vironostika HIV-1 Microelisa System, bioMerieux

b Fluorognost Sanochemia IFA

c Roche Cobas Amplicor HIV-1 Monitor Assay (ultra-sensitive to 50 copies/ml)

d Gen-Probe Procleix HIV-1 RNA Assay

e Bio-Rad HIV-1/HIV-2 plus O

f Genetic Systems HIV-1 Western blot

g Abbott HIVAB HIV-1/HIV-2 (rDNA) EIA

h Cambridge Biotech HIV-1 Western blot

i OraSure HIV-1 Western blot

Of the 72 persons classified as uninfected based on repeat confirmatory testing, 31 (43%) had OraQuick test-line appearance recorded; of these, 25 (81%) had a very faint test line (24 oral, 1 whole blood), 2 (7%) had a faint line (both oral), and 4 (13%) had a reddish test line (1 whole blood, 3 oral).

#### HIV-1 infected (True-positive rapid test)

Of the 17 persons classified as infected, 12 (71%) had a whole blood rapid test and 5 (29%) had an oral fluid rapid test.

Of the 17 persons with repeat confirmatory testing who were classified as HIV-1 infected, 15 (88%) had an initially indeterminate WB. Thirteen (76.5%) had initial confirmatory tests performed on oral fluid. Of these 13, 8 (62%) were EIA negative and 2 (15%) were WB negative (Table 2). Four persons who had an initial negative EIA and indeterminate WB on oral fluid had a repeatedly reactive EIA and positive WB on serum performed 1 to 8 days after the initial confirmatory test (Table 2). Of the 4 persons whose initial confirmatory specimen was serum, 1 of 4 (25%) tested EIA-negative, and 4/4 tested either IFA or WB indeterminate at the local laboratory. Of the 17 persons classified as HIV-infected, 3 (18%) were classified based on the detection of HIV-1 RNA following an indeterminate Western blot (Table 2). Of the 17 persons classified as infected, 5 (29%) had appearance of the OraQuick test line recorded: 2 (40%) had very faint test lines (1 oral-fluid, 1 whole blood) and 3 (60%) had a reddish test line (1 whole blood, 2 oral fluid).

**Table 2:** Test results for 17 HIV-infected persons with reactive rapid test results initially confirmed as either negative or indeterminate on Western blot or by indirect immunofluorescence, 17 health departments, 11 August 2004 to 31 December 2005.

	Initial Discordant Results			Repeat Confirmatory Results				
Oraquick specimen type	Confirmatory specimen type	EIA	Confirmatory test and result	Days after first confirmatory test	Confirmatory specimen type	EIA	WB/IFA result	Viral load copies/ml
Oral	Oral	Neg^a^	WB Indet^b^ gp120, gp160	4	Serum	Pos^c^	WB Pos^d^	ND
Oral	Oral	Neg^a^	WB Indet^b^ p24	8	Serum	Pos^a^ [Pos]	IFA Pos^e^ [WB Pos]^f^	ND
Oral	Oral	Neg^a^	WB Indet^b^ p24	28	Serum	Pos^a^ [Pos]	IFA Pos^e^ [WB Pos]^f^	ND
Oral	Oral	Neg^a^	WB Neg^b^	42	Serum	Neg^a^	WB Indet^f^ gp160* IFA Neg^e^	Detectable^g^
Oral	Oral	Neg^a^	WB Indet^b^ P24	–	–	ND	ND	>700,000^h^
Blood	Oral	Neg^a^	WB Indet^b^ p17, p24	1	Serum	Pos^a^ [Pos]	IFA Pos^e^ [WB Pos]^f^	ND
Blood	Oral	Neg^a^	WB Indet^b^ p24	6	Serum	Pos^c^ [Pos]	WB Pos^d^ [WB Pos]^f^	ND
Blood	Oral	Pos^a^	WB Indet^b^ p24	14	Oral	Pos^a^	WB Pos^b^	ND
Blood	Oral	Pos^a^	WB Indet^b^ p24, p66, gp120*, gp160*	14	Serum	Pos^a^,^i^,^j^ [Pos]	WB Pos^d^ [Pos]^f^	ND
Blood	Oral	Pos^a^	WB Indet^b^ p24	14	Serum	Pos^c^	WB Pos^d^	>20,000^g^
Blood	Oral	Pos^a^	WB Indet^b^ p24, gp160*	23	Serum	Pos^c^	WB Pos^d^	ND
Blood	Oral	Pos^a^	WB Indet^b^ gp120, gp160	38	Oral	Pos^a^	WB Indet^b^ gp120, gp160	>500,000^k^
Blood	Oral	Neg^a^	WB Neg^b^	69	Oral	Pos^a^	WB Pos^b^	ND
Blood	Serum	Pos a,i,j[Pos]	WB Indet^d^ gp41*, gp120*, gp160* [Pos]^f^	19	Serum	Pos^i^,^j^ [Pos]	WB Ind^d^ P31*, gp41*, gp120*, gp160* [Pos]	ND
Blood	Serum	Neg^a^	WB Indet^d^ p18*	<60	Serum	Pos^a^	WB Pos^d^	ND
Blood	Serum	Pos^i^,^j^ [Pos]	WB Indet^b^ p17, p24, p31*, p51, p55, p66, gp120*, gp160* [Pos]^f^	63	Serum	Pos^a^,^i^,^j^ [Pos]	WB Pos^d^ [Pos]	ND
Blood	Serum	ND [Pos]	IFA Indet^e^ [Pos]^f^	17	Serum	Pos	IFA Indet^l^	ND

EIA = enzyme immunoassay, IFA = immunofluorescent assay, WB = Western blot, Neg = Negative, Pos = Positive, Indet = Indeterminate, ND = Not done

If test result not bracketed, it was conducted by local laboratory.

* Bands interpreted as equivocal

[ ] results reported by CDC lab where Genetic Systems HIV1/HIV2 Plus O and Genetic Systems HIV-1 Westen blot were used unless other test indicated

a Vironostika HIV-1 Microelisa System, bioMerieux

b Orasure HIV-1 Western blot

c Bio-Rad HIV-1/HIV-2 plus O

d Genetic Systems HIV-1 Western blot

e Fluorognost HIV-1 IFA

f Cambridge Biotech HIV-1 Western blot

g bDNA Versant HIV RNA Assay (conducted 52 days after initial discordant result-viral load not reported)

h Amplicor HIV-1 Monitor v1.5

i Genetic Systems rLAV EIA

j Multispot HIV-1/HIV-2 rapid test

k Unknown

l Repeat confirmatory test not done at CDC because initial Western blot found to be positive

### Failure to Have Repeat Confirmatory Testing

In univariate analysis, the following characteristics were associated (p<0.2) with increased risk of not having repeat confirmatory testing and were included in the multivariable model: having male-female sex (compared with male-male sex), not having a previous HIV test, and having a negative initial confirmatory result (compared with indeterminate) (Table 3). Not having a previous HIV test was removed from the model due to its high correlation with history of male-female sex. In multivariate analysis, having male-female sex (compared with male-male sex) was associated (p<0.05) with increased risk of not having repeat confirmatory testing.

**Table 3:** Demographic, risk, and initial test characteristics of 172 persons with reactive rapid HIV test result and negative or indeterminate confirmatory test and proportion without a repeat confirmatory test; 17 health departments, 11 August 2004 to 31 December 2005.^a^

	Did not have repeat confirmatory test n/N (%)	Univariate OR (95% CI)	Univariate p-value	Multivariate aOR (95% CI)	Multivariate p-value
**Sex**					
Female	24/45 (53.3)	1.0			
Male	59/127 (46.5)	0.76 (0.38, 1.50)	p = 0.428	–	
**Age Group**					
<33	38/84 (45.2)	1.0		–	
> = 33	43/85 (50.6)	1.24 (0.68, 2.27)	p = 0.486		
**Race/Ethnicity**					
White non-Hispanic	35/78 (44.9)	1.0			
Black non-Hispanic	28/53 (52.8)	1.38 (0.68, 2.77)	p = 0.372	–	
Other non-Hispanic	9/17 (52.9)	1.38 (0.48, 3.96)	p = 0.546		
Hispanic	10/22 (45.5)	1.02 (0.40, 2.65)	p = 0.961		
**Sexual Behavior**					
Male-male sex	22/65 (33.9)	1.0		1.0	
Male-female sex	59/103 (57.3)	2.62(1.38, 5.00)	p = 0.003*	2.55 (1.33, 4.89)^a^	p = 0.005*
**Injection drug use**					
No injection drug use	68/143 (47.6)	1.0		–	
Injection drug use	13/25 (52.0)	1.20 (0.51, 2.80)	p = 0.681		
**Previously HIV Tested**					
Yes	55/127 (43.3)	1.0		–	
No	27/41 (65.9)	2.52 (1.21, 5.26)	p = 0.014*		
**Initial confirmatory specimen**				–	
Serum/plasma	66/132 (50.0)	1.35 (0.66, 2.76)	p = 0.407		
Oral Fluid	17/40 (42.5)	1.0			
**Initial rapid HIV test context**				–	
Confidential	50/101 (49.5)	1.0			
Anonymous	31/69 (44.9)	0.83 (0.45, 1.54)	p = 0.557		
**Initial confirmatory test**					
Negative	69/134 (59.5)	1.82 (0.87, 3.82)	p = 0.113	1.89 (0.87, 4.10)^b^,	p = 0.108
Indeterminate	14/38 (36.8)	1.0		1.0	
**Site type**					
Non-traditional site (Outreach/prison/other)	16/36 (44.4)	1.0		–	
Traditional clinic site	63/128 (49.2)	1.21 (0.58, 2.55)	p = 0.613		

aOR, adjusted odds ratio; CI, confidence interval.

* Statistically significant

a adjusted for initial confirmatory test result

b adjusted for sexual behavior

### Reasons for not obtaining repeat confirmatory test specimens

Thirteen of eighteen health departments had at least one discordant case that did not have repeat confirmatory testing. Principal investigators from these health departments gave the following reasons for not repeating confirmatory testing on discordant clients: unable to locate clients (6/13 (46%) health departments), client did not return for testing (5/13 (39%) health departments), client refused (1/13 (8%) health departments) and unknown (3/13 (23%) health departments).

## Discussion

Despite national guidelines in the United States (U.S.) recommending repeat confirmatory testing for persons with a reactive rapid test result and negative or indeterminate confirmatory test result, only half of the persons with discordant test results had a repeat confirmatory test during post-marketing surveillance [9], [10]. The importance of repeat confirmatory testing is clear given our finding that overall nearly one in five persons with discordant test results who underwent repeat confirmatory testing were found to be HIV-infected, including over half of those whose initial confirmatory test was WB/IFA indeterminate. In addition, repeat confirmatory testing identified two HIV-infected persons whose initial Western blot results were negative. Repeat confirmatory testing is particularly important for persons with discordant HIV test results who were initially confirmed with an oral fluid specimen: over half of persons who tested rapid test reactive who had a negative or indeterminate WB performed on oral fluid were found to be HIV-infected. Based on these findings and given the higher sensitivity of blood tests compared with oral fluid tests, testing with blood for the initial and repeat confirmatory tests following a reactive rapid test is preferable, when possible. Our findings on the high proportion of persons with discordant test results who do not have repeat confirmatory testing and the prevalence of HIV infection among persons with discordant rapid test results suggest that some HIV-infected persons with discordant results may be misinformed that they are *uninfected* based on the results of a single, initial confirmatory test result that is negative. These findings underscore the need for state and local rapid HIV testing programs to work with persons with discordant rapid HIV test results to ensure that they have repeat confirmatory testing.

Persons with discordant rapid HIV test results who had male-female sex were at higher risk for not having repeat confirmatory testing. It is possible that some of these testers were perceived to be of lower HIV risk than men who have sex with men, so their rapid test result was viewed as false positive based on the initial negative or indeterminate confirmatory test. Also, principal investigators of participating health departments indicated that not being able to locate clients or clients not returning for testing were the primary reasons for clients not having repeat confirmatory testing. A significant proportion (37%) of those without a repeat confirmatory test tested anonymously so they could not be reached for further testing. To increase repeat confirmatory testing, testing staff should encourage all persons with discordant HIV test results to have repeat confirmatory testing done at the visit during which they receive their initial negative or indeterminate confirmatory results. However, additional repeat testing may be necessary to allow sufficient time for seroconversion [18].

Given the well-publicized clusters of excess false-positive oral fluid rapid test results, some counseling and testing staff may also have been less concerned about recommending repeat confirmatory testing for clients who initially had an unconfirmed reactive oral fluid rapid test result [4]–[7]. Reactive rapid test results that do not confirm positive should not be presumed to be false positive. Of those with discordant test results determined to be HIV-infected, at least two had OraQuick test lines reported to be very faint (one whole blood and one oral fluid). Upon seeing any OraQuick test line, including those which are very faint, it is necessary to pursue confirmatory testing and repeat confirmatory testing (if warranted) and not assume that the rapid test is false positive.

Of the HIV-infected persons with initially discordant confirmatory test results, four persons with an indeterminate WB on oral fluid had a positive WB on serum less than 9 days after the initial confirmatory test. In addition, compared with those who initially confirmed with serum, proportionally more persons with reactive rapid test results who initially confirmed WB negative or indeterminate on oral fluid were found to be HIV-infected on follow-up. This is likely due to the decreased sensitivity of the oral fluid test relative to serum, and it underscores the need to use serum or plasma for confirmatory tests when possible due to the lower concentration of antibody in oral fluid compared with serum or plasma [9]–[13]. We were encouraged to find that among those clients who underwent repeat confirmatory testing, most did so with a blood specimen.

Rapid HIV test providers should also be aware that some HIV-infected clients with discordant test results may take time to fully seroconvert, even when repeat confirmatory tests are performed on serum or plasma. Of note, one initially discordant rapid test client had negative results for both a serum EIA and IFA performed 42 days *after* a reactive oral-fluid rapid test result. In the absence of an indeterminate WB conducted at the time of the negative EIA and negative IFA and a detectable NAAT conducted 10 days later, this apparently HIV-infected person would have been informed that he was not infected according to current U.S. confirmation guidelines [9], [18]. The possibility exists, though, that this infection was acquired after the initial reactive rapid test. Additionally, two other persons with discordant rapid test results who were classified as HIV-infected had an indeterminate repeat WB and a detectable NAAT. In these three cases, NAAT provided further information about infection status beyond WB test results. Since the publication of rapid test confirmation recommendations in 2003, one NAAT has been approved by the FDA for HIV diagnostic confirmation [19]. Thus, NAAT should be considered in addition to WB or IFA for repeat confirmatory testing to help resolve the infection status of persons with discordant rapid HIV test results. It's important to note that a detectable NAAT may indicate infection, though an undetectable result does not verify a lack of infection [19].

Among those with discordant test results who had repeat confirmatory tests, most (80%), were found to be HIV uninfected. Of those classified as HIV uninfected, twelve persons who did not have evidence of HIV infection based on negative EIA, IFA, and NAAT results at their repeat test had an indeterminate repeat WB result. Only one of the twelve developed a major HIV band (p24) during follow-up, which can occur in uninfected persons [16]. This person had a non-reactive EIA on repeat testing, which provided evidence that they were likely uninfected, though a repeat WB conducted on serum or NAAT on plasma may have provided more information. Because of the high prevalence of indeterminate WB results among persons who are not HIV-infected, the use of other confirmatory assays should be considered [17].

This surveillance project was subject to some limitations which should be mentioned. Local laboratories utilized a variety of EIA, WB and NAAT tests which have varying sensitivities and specificities, and repeat tests were conducted at varying intervals after the initial discordant test. However, all remnant serum or plasma specimens with sufficient volume sent to CDC were uniformly tested with a third-generation IgM-sensitive EIA, WB, and NAAT. Though the ultimate HIV infection classification of cases with repeat confirmatory testing appears to be correct, it is possible that the use of pooled NAAT on serum (an off label use) could have missed some early infections and resulted in misclassification. Additionally, some persons with an indeterminate repeat test result classified as uninfected could have been misclassified because of relatively short retesting intervals (i.e. insufficient time for seroconversion). However, of the 6 persons whose indeterminate repeat test occurred less than the median follow-up of 24 days, 3/3 were IFA negative and 3/3 were NAAT negative. An additional limitation of the surveillance project is potential under-reporting of discordant cases, though CDC staff regularly contacted health departments to gauge whether all discordant cases had been reported. Finally, another limitation is that the tests utilized are limited to those available in the U.S. and the testing guidelines mentioned are specific to the U.S., so results may not be generalizable to other countries.

The findings from this post marketing surveillance project underscore the need for rapid HIV testing programs to work with persons with reactive rapid tests and negative or indeterminate confirmatory test results to ensure that they have repeat confirmatory testing on a new specimen obtained during a follow-up visit. Due to the lower sensitivity of the WB performed on oral fluid, confirmatory testing following a reactive rapid test should be conducted using serum or plasma, when possible.

## References

[1] CDC (2002). Notice to Readers: Approval of a New Rapid Test for HIV Antibody.. MMWR.

[2] CDC CLIA certificate of waiver fact sheet. Accessed Aug 2007.. http://www.cdc.gov/rapid_testing/materials/roltCLIA.htm.

[3] (2004). OraQuick Advance Rapid HIV-1/2 Antibody Test package insert..

[4] CDC (2005). Supplemental Testing for Confirmation of Reactive Oral Fluid Rapid HIV Antibody Tests.. MMWR.

[5] Delaney KP, Branson BM, Uniyal A, Kerndt PR, Keenan PA (2006). Performance of an Oral Fluid Rapid HIV 1/2 Test: Experience from Four CDC Studies. AIDS.

[6] Jafa K, Patel P, MacKellar DA, Sullivan PS, Delaney KP (2007). Investigation of False Positive Results with an Oral Fluid Rapid HIV-1/2 Antibody Test.. PLoS ONE.

[7] Wesolowski LG, MacKellar DM, Facente SN, Dowling T, Ethridge SF (2006). Post-Marketing Surveillance of OraQuick Whole-Blood and Oral-Fluid Rapid HIV Testing AIDS.

[8] Stekler J, Wood RW, Swenson PD, Golden M (2007). Negative Rapid HIV Antibody Testing during Early HIV Infection.. Ann Intern Med.

[9] CDC (2007). Quality Assurance Guidelines for Testing Using Rapid HIV Antibody Tests Waived under the Clinical Laboratory Improvement Amendments of 1988.. http://www.cdc.gov/hiv/topics/testing/resources/guidelines/pdf/QA_Guidlines_OraQuick.pdf.

[10] CDC (2004). Notice to readers: protocols for confirmation of reactive rapid HIV tests. MMWR 53: 221-2. OraSure HIV-1 Western Blot Kit package insert.. MMWR.

[11] OraSure HIV-1 Western Blot Kit package insert.

[12] Gallo D, George JR, Fitchen JH, Goldstein AS, Hindahl MS (1997). Evaluation of a system using oral mucosal transudate for HIV-1 antibody screening and confirmatory testing.. JAMA..

[13] Granade TC, Phillips SK, Parekh B, Gomez P, Kitson-Piggott W (1998). Detection of antibodies to human immunodeficiency virus type 1 in oral fluids: a large-scale evaluation of immunoassay performance.. Clinical and Diagnostic Laboratory Immunology.

[14] Soto-Ramirez LE, Hernandez-Gomez L, Sifuentes-Osornio J, Barriga-Angulo G, Duarte de Lima D (1992). Detection of specific antibodies in gingival crevicular transudate by enzyme-linked immunosorbent assay for diagnosis of human immunodeficiency virus type 1 infection.. J Clin Microbiol..

[15] CDC (2006). Rapid HIV Test Distribution-United States, 2003–2005.. MMWR.

[16] CDC (1989). Interpretation and use of the Western blot assay for serodiagnosis of human immunodeficiency virus type 1 infections.. MMWR.

[17] Celum CL, Coombs RW, Lafferty W, Inui TS, Louie PH (1991). Indeterminate human immunodeficiency virus type 1 western blots: seroconversion risk, specificity of supplemental tests, and an algorithm for evaluation.. J. Infect Dis.

[18] CDC (2001). Revised Guidelines for HIV Counseling, Testing, and Referral.. MMWR.

[19] (2006). Aptima HIV-1 RNA Qualitative Assay Package Insert..

